# Circular RNA hsa_circ_0057452 facilitates keloid progression by targeting the microRNA-1225-3p/AF4/FMR2 family member 4 axis

**DOI:** 10.1080/21655979.2022.2084460

**Published:** 2022-06-15

**Authors:** Hu Gao, Zhen Hu, Xiangming Zhang

**Affiliations:** a Wound Repair & Rehabilitation Centre, Tongren Hospital of Wuhan University (Wuhan Third Hospital), Wuhan, Hubei, China; b Department of Dermatology, Tongren Hospital of Wuhan University (Wuhan Third Hospital), Wuhan, Hubei, China

**Keywords:** Hsa_circ_0057452, miR-1225-3p, AFF4, keloid, KF

## Abstract

The circular RNA, hsa_circ_0057452, is highly expressed in keloids, but its specific mechanism of action remains unknown. The levels of hsa_circ_0057452, microRNA (miR)-1225-3p, and AF4/FMR2 family member 4 (AFF4) in keloid tissues and keloid fibroblasts (KFs) were determined using quantitative reverse transcription-polymerase chain reaction. Changes in KFs viability, proliferation, apoptosis, and migration were investigated using the cell counting kit-8, bromodeoxyuridine, flow cytometry, and Transwell assays. Luciferase, RNA immunoprecipitation, and RNA pull-down assays were performed to identify the binding relationship among hsa_circ_0057452, miR-1225-3p, and AFF4. We found that hsa_circ_0057452 and AFF4 expression levels were upregulated, whereas miR-1225-3p expression levels were downregulated in keloids. Knockdown of hsa_circ_0057452 or AFF4 suppressed the viability, proliferation, and migration of KFs and induced apoptosis, whereas hsa_circ_0057452 overexpression and miR-1225-3p knockdown showed the opposite trend. Furthermore, hsa_circ_0057452 affected the biological behavior of KFs by releasing AFF4 via sponging of miR-1225-3p. Therefore, our results show that hsa_circ_0057452 promotes keloid progression by targeting miR-1225-3p and regulating AFF4 levels.

## Highlights

- Expression levels of hsa_circ_0057452 and AFF4 are upregulated, while those of miR-1225-3p are downregulated in keloids.
- Knockdown of hsa_circ_0057452 or AFF4 suppresses the KFs viability, proliferation, and migration, while inducing apoptosis.
- Hsa_circ_0057452 overexpression and miR-1225-3p interference promote the KFs viability, proliferation, and migration, while suppressing apoptosis.
- Hsa_circ_0057452 releases AFF4 by sponging miR-1225-3p.

## Introduction

Keloids are formed as a pathological response to skin lesions that disproportionately affect the skin color, mostly causing itching and pain, and reducing the quality of life [1,2]. Currently, the most common treatment methods for keloids are laser therapy, radiotherapy, surgical resection, cryotherapy, and topical steroid therapy [3,4]. However, these treatment methods are not yet fully effective in inducing keloid tissue degeneration or in preventing their postoperative recurrence [5]. Additionally, genetic factors are involved in the progression of keloids [6]. Therefore, the search for valuable biomarkers may aid in the development of effective novel therapies for keloids.

Circular RNAs (circRNAs) are covalently closed single-stranded RNAs whose 3′ and 5′ ends of exons are tightly linked in various highly conserved species [7]. Due to the development of high-throughput sequencing techniques and bioinformatics analysis, circRNAs have been found to play a crucial role in various biological processes, including cell survival, migration, and apoptosis [8]. Additionally, circRNAs have various post-transcriptional functions, including serving as miRNA sponges to the regulate target gene transcription and translation [9]. For example, circRNA-5692 induces the DAB2 interacting protein by reducing the microRNA (miR)-328-5p expression levels, thereby inhibiting the malignant behavior of hepatocellular carcinoma cells and tumor growth in vivo [10]. circRNA Rap guanine nucleotide exchange factor 5 predicts the poor invasiveness and long overall survival of patients with renal cell carcinoma and inhibits the survival and metastasis of cancer cells via the miR-27a-3p/thioredoxin interacting protein pathway in vitro and in vivo [11]. circ-ZNF609 promotes cervical cancer progression by modulating the miR-197-3p/E2F transcription factor 6 axis as an oncogene [12]. Hsa_circ_0057452, a lesser known circRNA, is confined to the keloids. Shi et al. [13] carried out Gene Ontology and Kyoto Encyclopedia of Genes and Genomes analysis to reveal that hsa_circ_0057452 expression levels were significantly upregulated in keloid tissues than in normal skin tissues. This finding suggests that hsa_circ_0057452 may play an important role in the development of keloids. However, the role of hsa_circ_0057452 as a sponge in keloids has not yet been fully elucidated.

Some miRNAs are associated with the growth, proliferation, and differentiation of keloid fibroblasts (KFs). For example, upregulation of miR-4417 expression inhibits the invasion, migration, and proliferation of KFs, while facilitating apoptosis [14]. Overexpression of miR-203 inhibits the malignant behavior and extracellular matrix production in KFs [15]. miR-1225-3p inhibits tumor growth by inhibiting the cell proliferation and migration [16]. Additionally, AF4/FMR2 family member 4 (AFF4) is a scaffold protein that binds to transcription factors and induces gene transcription via elongation and chromatin remodeling [17]. However, the effects of miR-1225-3p and AFF4 on KFs remain unclear.

This study aimed to investigate the functional role of hsa_circ_0057452 in keloid growth and clarify the key role of the hsa_circ_0057452/miR-1225-3p/AFF4 axis in the growth regulation of KFs. We hypothesized that hsa_circ_0057452 may participate in the biological behavior of KFs by releasing AFF4 via sponging of miR-1225-3p. This may provide a promising strategy for keloid treatment.

## Methods

### Tissue samples

Keloid and normal skin tissues matched with keloids ≥10 cm were obtained from 34 patients with keloids recruited from the Tongren Hospital of Wuhan University (Wuhan Third Hospital). Pathologists confirmed the pathological features of the samples. This study was approved by the Ethics Committee of Tongren Hospital of Wuhan University (Wuhan Third Hospital, approval number: KY2022-025), and written informed consent was obtained from all participants. The clinicopathological features of all patients are summarized in Supplementary Table S1.

### Cell collection and culture

Keloid tissues, removed from the subcutaneous adipose tissue and matched normal skin tissues, were eliminated using trypsin digestion to obtain KFs and normal fibroblasts (NFs). Briefly, the tissues were washed with the dispase II solution (Sigma Aldrich, USA) to remove the epidermis and incubated for 4 h at 37°C. The tissues were then cut into small pieces of 1 cm^3^ and digested with 0.05% trypsin (10 min each time). After digestion, the digested liquid was centrifuged and placed in Dulbecco’s modified Eagle’s medium (DMEM) medium containing 10% phosphate-buffered saline at 37°C and CO_2_%.

### Cell transfection

miR-1225-3p inhibitor and inhibitor negative control (NC) were purchased from SwitchGear Genomics (USA). Small interfering RNA (siRNA) for hsa_circ_0057452 (si-circ-1 and si-circ-2), siRNA for AFF4 (si-AFF4), siRNA non-targeting control (si-NC), hsa_circ_0057452 overexpression vector (OE-circ), and OE-NC were purchased from RiBobo (China). When KFs reached 80% confluence, 75 nM of inhibitor, 50 nM of siRNA or 2 μg/mL of overexpression RNA were transfected into the cells using Lipofectamine 2000 reagent (Invitrogen, USA). After transfection for 48 h, transfection efficiency was measured using quantitative reverse transcription-polymerase chain reaction (qRT-PCR). The siRNA sequences used in this study are listed in Supplementary Table S2.

### qRT-PCR

miRNAs extracted using the miRNeasy Mini kit (Qiagen, China) were transcribed using the TaqMan MicroRNA Reverse Transcription Kit (Applied Biosystems) and miRNA-specific stem-loop primers. Subsequently, a TaqMan MicroRNA Assay (Applied Biosystems) was used to measure the miR-1225-3p levels with the help of Applied Biosystems 7500 (Thermo Fisher Scientific). U6 small nuclear RNA (U6) served as the control, using the 2^−ΔΔCt^ method [18].

The Norgen Biotek Total RNA Purification Kit (PA, USA) was used to extract the total RNA. cDNA was synthesized using the PrimeScript RT kit (Takara, Japan), followed by qPCR using the SYBR Green PCR Master Mix (Takara). Glyceraldehyde-3-phosphate dehydrogenase (GAPDH) was used as the negative control. The primer sequences are listed in Table 1.

**Table 1.** Primer sequences used in this research

Gene	Sequences of primers(5’-3’)
circ_0057452	Forward primer:GTATGCCTGGAAAACCTGGA
	Reverse primer:AGGGCCTTCAAGACCTTTGT
miR-1225-3p	Forward primer:GCGGCGGTGAGCCCCTGTGCCG
	Reverse primer:ATCCAGTGCAGGGTCCGAGG
AFF4	Forward primer:AAAGGCCAGCATGGATCAGAA
	Reverse primer:GTGATTTGGAGCGTTGATGTTC
TRAM1	Forward primer:5’-AATTCCTGCCCTCTTTCTCTCT-3’
	Reverse rimer:5’-TGCTCAGCAACATTACACAAGG-3’
KIF3B	Forward primer:ATCCTGGAGCAGAAACGACAGG
	Reverse primer:GTTCCAAGGTCTCCTCATCTCG
GAPDH	Forward primer:AGCCACATCGCTCAGACAC
	Reverse primer:GCCCAATACGACCAAATCC
U6	Forward primer:CGCTTCGGCAGCACATATACTA
	Reverse primer:CGCTTCACGAATTTGCGTGTCA

### RNase R treatment

RNase R (Epicenter Technologies, USA) was used to digest the total RNA from KFs. RNA (2 μg) was incubated with 4 U/μg RNase R for 30 min at 37°C. Then, the incubated RNA was purified using the RNEasy Minelute Cleanup Kit (Qiagen, USA), and hsa_circ_0057452 or its linear transcript (linear hsa_circ_0057452) levels were measured using qRT-PCR [19].

### RNA-fluorescence in situ hybridization (FISH)

FISH was performed according to the manufacturer’s instructions (GenePharma, Shanghai, China). KFs were collected, fixed with 4% paraformaldehyde, and treated with 70, 85, and 100% alcohol for 5 min to dehydrate. Hybridization was performed using the hsa_circ_0057452 probe. After hybridization, the samples were washed with 50% formamide (2 × SSC). Cell nuclei were stained with 4′,6-diamidino-2-phenylindole. The subcellular distribution of hsa_circ_0057452 in KFs was observed using a confocal laser scanning microscope (Olympus FV1000) [20].

### Cell counting kit-8 (CCK-8) assay

The CCK-8 cell proliferation test kit (Dojindo, Japan) was used to estimate the cell viability, according to the manufacturer’s instructions. Transfected KFs were collected and placed in a 48-well plate (1 × 10^4^/mL) and maintained in a humidified chamber at 37°C. Then, 10 μL of CCK-8 solution was added to each well at 0, 12, 24, and 48 h. After incubation for 4 h, the optical density was measured at 450 nm using a microplate reader (Bio-Rad Laboratories, USA) [21].

### Bromodeoxyuridine (BrdU) assay

KFs (5 × 10^3^ cells/well) were seeded in a 96-well plate and cultured for 24 h. Enzyme-linked immunosorbent assay (BrdU kit; Beyotime, China) was used to analyze the incorporation of BrdU during DNA synthesis, according to the manufacturer’s instructions. Absorbance was measured using a microplate reader at 450 nm [22].

### Apoptosis assay

Annexin V-fluorescein isothiocyanate (FITC)-propidium iodide (PI) Apoptosis Detection Kit (KeyGen Biotech, China) was used to analyze the apoptosis rate of KFs. Briefly, the cells were digested with trypsin, centrifuged at 250 × *g* for 5 min, and resuspended in a binding buffer. Then, 5 μL of Annexin V-FITC and 5 μL of PI were added to the cell suspension and incubated in the dark for 15 and 5 min at 25°C, respectively. Subsequently, the apoptotic rates were measured using flow cytometry (BD FACSCalibur, USA) [21].

### Transwell assay

Cells (5 × 10^4^) resuspended in DMEM were injected into the upper chamber of the Transwell insert (Corning, USA), and the complete medium was placed in the lower chamber. After 24 h, the migrated cells in the lower chamber were fixed with paraformaldehyde, stained with crystal violet, and photographed with an optical microscope (Olympus, Japan) [23].

### Luciferase reporter assay

The wild-type sequence of hsa_circ_0057452 or AFF4 (circ-WT or AFF4-WT), containing the miR-1225-3p binding site, was synthesized and cloned into the psiCHECK-2 luciferase vector (Promega, USA). The mutant reporting vectors (circ-MUT or AFF4-MUT) of hsa_circ_0057452 or AFF4 were synthesized by Sangon Biotech (China). The reporter vector was transfected into the cells transfected with miR-1225-3p mimic/mimic-NC using Lipofectamine 2000 (Invitrogen). After 48 h, luciferase activity was measured using a dual-luciferase reporter assay kit (Promega, USA) [24].

### RNA immunoprecipitation (RIP) assay

This analysis was performed using an RNA binding protein immunoprecipitation kit (Millipore, USA). Cells were lysed using the RNA lysis buffer for 30 min and co-incubated with the RIP binding buffer having magnetic beads coated with 5 µg of anti-RIP-AGO2 antibody (Millipore) or IgG (Millipore) for 4 h at 4°C. Enrichment of hsa_circ_0057452 and miR-1225-3p were measured using qRT-PCR [25].

### RNA pull-down assay

Cells treated with biotin-labeled miR-1225-3p (Bio-miR-1225-3p) or Bio-NC (Sangon, China) were lysed using a lysis buffer (Promega). Dynabeads M-280 Streptavidin beads (Life Technologies, USA) were blocked with RNase-free bovine serum albumin (BSA) and yeast tRNA (Sigma-Aldrich) for 30 min at 4°C. Subsequently, the cell lysates were incubated with blocked beads at 25°C for 2 h, followed by qRT-PCR analysis [26].

### Western blotting assay

Proteins were extracted using a radioimmunoprecipitation assay (Boster, China), and protein content was estimated using the bicinchoninic acid assay (Boster). They were electrophoresed in 10% sulfate-polyacrylamide gel. Subsequently, the proteins were transferred onto polyvinylidene fluoride membranes, washed with Tris-buffered saline with Tween 20, and blocked with 5% BSA blocking buffer at 37°C for 2 h. Then, primary antibodies, AFF4 (ab103586, Abcam, UK) and GAPDH (ab8245, Abcam), were incubated with the membranes overnight at 4°C, prior to incubation with secondary antibody (ab6721, Abcam) for 1 h at 37°C. The ECL detection kit (Yeasen, China) and ImageJ software (Version 1.48; NIH, USA) were used to visualize and determine the protein levels [27].

### Statistical analysis

Data from at least three independent experiments are represented as the mean ± standard deviation using GraphPad Prism Software (La Jolla, USA). Comparisons were made using the Student’s t-test and one-way analysis of variance. Differences were considered statistically significant at P < 0.05.

## Results

This study aimed to investigate the functional role of hsa_circ_0057452 in keloid growth. We hypothesized that hsa_circ_0057452 could facilitate the malignant behavior of KFs. In this study, we found that hsa_circ_0057452 expression levels were remarkably upregulated in keloids. Moreover, hsa_circ_0057452 adsorbed miR-1225-3p to further upregulate AFF4 expression levels to facilitate keloid progression.

### Silencing hsa_circ_0057452 inhibits the survival and migration of KFs, and facilitates their apoptosis

Expression levels of hsa_circ_0057452 in keloid tissues (K) were upregulated approximately 2.3-fold compared to those in the normal tissues (NS; P < 0.0001; Figure 1(a)). Similarly, the levels of hsa_circ_0057452 in the isolated and cultured primary KFs were approximately 4.3 times than those in NFs (P = 0.0001; Figure 1(b)). In addition, the circular stability of hsa_circ_0057452 was investigated after RNase R treatment. We observed that the linear hsa_circ_0057452 levels (P < 0.0001) were downregulated by approximately 60% in the RNase R^+^ group compared with those in the RNase R^−^ group, while there were no significant changes in the hsa_circ_0057452 levels (P = 0.5432; Figure 1(c). Moreover, the subcellular localization of hsa_circ_0057452 was evaluated using FISH, and it was found that hsa_circ_0057452 was expressed mainly in the cytoplasm (Figure 1(d)). Based on these results, a specific hsa_circ_0057452 siRNA was delivered into the KFs. Transfection data revealed that hsa_circ_0057452 expression levels in the si-circ-1 (P < 0.0001) and si-circ-2 (P < 0.0001) groups at 48 h decreased by 75 and 60%, respectively, compared to those in the si-NC group (Figure 1(e)). Functional analysis was performed to explore the effects of hsa_circ_0057452 expression on KFs viability, apoptosis, and migration. CCK-8 assay showed that in contrast to the si-NC group, cell viability in si-circ-1 and (P < 0.0001, at 48 h) si-circ-2 (P < 0.0001, at 48 h) groups was reduced by about 45 and 30%, respectively (Figure 1(f)). BrdU assay revealed approximately 50 and 40% decrease in cell proliferation in si-circ-1 (P = 0.0006) and si-circ-2 (P = 0.0035) groups, respectively, compared to that in the si-NC group (Figure 1(g)). Flow cytometry revealed that the si-circ-1 (P < 0.0001) and si-circ-2 (P < 0.0001) groups enhanced the apoptosis rate by 3.1-fold and 2.4-fold, respectively, compared to the si-NC group (Figure 1(h)). In addition, transwell assays showed that the knockdown of hsa_circ_0057452 in the si-circ-1 (P < 0.0001) and si-circ-2 (P < 0.0001) groups reduced the cell migration by approximately 75 and 60%, respectively, compared to the si-NC group (Figure 1(i)).

**Figure 1.** Silencing hsa_circ_0057452 inhibits the survival and migration of KFs, and facilitates their apoptosis. (a) The relative RNA levels of hsa_circ_0057452 were evaluated by qRT-PCR between keloid tissues (K, n = 34) and normal skin (NS, n = 34). **P < 0.001. (b) The relative RNA levels of hsa_circ_0057452 were evaluated by qRT-PCR between KFs and NFs. **P < 0.001 vs. NFs. (c) The stability of hsa_circ_0057452 were evaluated by RNase R treatment in KFs. **P < 0.001 vs. RNase R-. (d) hsa_circ_0057452 subcellular localization was evaluated by FISH analysis in KFs. (e) The silent efficiency of hsa_circ_0057452 was evaluated by qRT-PCR in KFs transfected with si-NC, si-circ-1 and si-circ-2, respectively. (f) CCK-8 assays were performed to assess the viability in KFs transfected with the si-NC, si-circ-1 and si-circ-2, respectively. (g) BrdU assays were performed to assess the proliferation ability in KFs transfected with the si-NC, si-circ-1 and si-circ-2, respectively. (h) Cell apoptosis was examined using flow cytometry in KFs transfected with the si-NC, si-circ-1 and si-circ-2, respectively. (i) Transwell migration assays were applied for assessing the migration ability of KFs transfected with the si-NC, si-circ-1 and si-circ-2, respectively. **P < 0.001 vs. si-NC.

### Overexpression of hsa_circ_0057452 facilitates the survival and migration of KFs, and inhibits their apoptosis

Next, the hsa_circ_0057452 overexpression plasmid was delivered to KFs. qRT-PCR revealed that compared to the OE-NC group, the expression levels of hsa_circ_0057452 in the OE-circ group was upregulated by approximately 3.5-fold (P < 0.0001; Figure 2(a)). CCK-8 and BrdU assays showed that cell viability (P < 0.0001, at 48 h) and proliferation (P = 0.0073) in the OE-circ group were higher than those in the OE-NC group (Figure 2(b,c)). Flow cytometry exhibited that the OE-circ group had a 65% (P = 0.0005) lower rate of apoptosis than the OE-NC group (Figure 2(d)). In addition, Transwell assays revealed that cell migration was about 1.3 times (P = 0.0042) higher in the OE-circ group than in the OE-NC group (Figure 2(e)).

**Figure 2.** Overexpression of hsa_circ_0057452 facilitates the survival and migration of KFs, and inhibits their apoptosis. (a) The overexpressed efficiency of hsa_circ_0057452 was evaluated by qRT-PCR in KFs transfected with OE-NC and OE-circ, respectively. (b) CCK-8 assays were performed to assess the viability in KFs transfected with the OE-NC and OE-circ, respectively. (c) BrdU assays were performed to assess the proliferation ability in KFs transfected with the OE-NC and OE-circ, respectively. (d) Cell apoptosis was examined using flow cytometry in KFs transfected with the OE-NC and OE-circ, respectively. (e) Transwell migration assays were applied for assessing the migration ability of KFs transfected with the OE-NC and OE-circ, respectively. **P < 0.001 vs. OE-NC.

### miR-1225-3p is sponged by hsa_circ_0057452

As shown in Figure 3(a), a query on the sharing website showed that miR-1225-3p contained hsa_circ_0057452 binding sites. Analysis of luciferase activity revealed that circ_0057452-WT combined with miR-1225-3p mimic reduced the KFs luciferase activity by approximately 50% (P < 0.0001) compared to circ_0057452-WT combined with miR-NC. (Figure 3(b)). It has been suggested that miR-1225-3p may bind to hsa_circ_0057452. Furthermore, RIP analysis confirmed that the enrichment levels of miR-1225-3p (P < 0.0001) and hsa_circ_0057452 (P < 0.0001) both increased in AGO2 compared to IgG (Figure 3(c)). Differential miR-1225-3p expression was detected using qRT-PCR, and the expression levels of miR-1225-3p in the K group were decreased by more than 70% (P < 0.0001) compared to those in the NS group (Figure 3(d)). Additionally, miR-1225-3p levels in KFs decreased by approximately 65% (P = 0.007) compared to those in NFs (Figure 3(e)). In conclusion, miR-1225-3p was underexpressed in keloids and sponged by hsa_circ_0057452.

**Figure 3.** miR-1225-3p is sponged by hsa_circ_0057452. (a) Schematic diagram of hsa_circ_0057452 and miR-1225-3p. (b) The relative luciferase activities were evaluated in HKFs after co-transfection with hsa_circ_0057452-WT or c hsa_circ_0057452-MUT and miR-1225-3p mimic or miR-NC, respectively. **P < 0.001 vs. miR-NC. (c) RIP assay was performed to examine the enrichment of hsa_circ_0057452 in keloid fibroblasts treated with RIP-AGO2 or RIP-IgG. **P < 0.001 vs. Anti-IgG. (d) The relative levels of miR-1225-3p were evaluated by qRT-PCR between keloid tissues (k) and normal skin (NS). **P < 0.001. (e) The relative levels of miR-1225-3p were evaluated by qRT-PCR between KFs and NFs. **P < 0.001 vs. NFs.

### miR-1225-3p is sponged by hsa_circ_0057452 to affect the malignant behavior of KFs

Next, we investigated functional changes in KFs induced by miR-1225-3p in cooperation with hsa_circ_0057452. Transfection efficiency analysis showed that si-circ transfection increased the level of miR-1225-3p by 3.5-fold compared to the si-NC group (P < 0.0001), and continued treatment with the miR-1225-3p inhibitor eased the upregulation of miR-1225-3p (Figure 4(a)). CCK-8 assay showed that cell viability was promoted in the si-circ + inhibitor group at 48 h in contrast to that in the si-circ + inhibitor-NC group (P < 0.0001, at 48 h; Figure 4(b)). BrdU showed that cell proliferation was facilitated in the si-circ + inhibitor group compared to the si-circ + inhibitor-NC group (P = 0.0344; Figure 4(c)). Flow cytometry revealed that the miR-1225-3p inhibitor reduced the apoptosis rate by approximately 50% compared to the si-NC group (P < 0.0001) and reversed the increase in apoptosis caused by si-circ (Figure 4(d)) In addition, the Transwell assay revealed that interference with miR-1225-3p promoted KF migration compared to the si-NC group (P < 0.0001) and partially eliminated migration inhibition caused by downregulation of hsa_circ_0057452 (Figure 4(e)).

**Figure 4.** miR-1225-3p is sponged by hsa_circ_0057452 to affect the malignant behavior of KFs. (a) The transfection efficiency of miR-1225-3p was evaluated by qRT-PCR in KFs transfected with si-circ or miR-1225-3p inhibitor. (b) CCK-8 assays were performed to assess the viability in KFs transfected with si-circ or miR-1225-3p inhibitor. (c) BrdU assays were performed to assess the proliferation ability in KFs transfected with si-circ or miR-1225-3p inhibitor. (d) Cell apoptosis was examined using flow cytometry in KFs transfected with si-circ or miR-1225-3p inhibitor. (e) Transwell migration assays were applied for assessing the migration ability of KFs transfected with si-circ or miR-1225-3p inhibitor. *P < 0.05, **P < 0.001 vs. si-NC; ##P < 0.001 vs. si-circ+inhibitor-NC.

### miR-1225-3p targets AFF4

To explore the downstream targets of miR-1225-3p, we used miRDB to forecast the miR-1225-3p target genes, and the top five genes in the miRDB database are listed in Supplementary Table S3. RNA pull-down was utilized to evaluate the binding of miR-1225-3p to mRNA. The enrichment levels of translocation associated membrane protein 1 (TRAM1), AFF4, kinesin family member 3 B (KIF3B), melanin-concentrating hormone receptor 1 (MCHR1), and BICD family like cargo adaptor 2 (BICDL2) on Bio-miR-1225-3p were 5.2 times (P = 0.0276), 91 times (P < 0.0001), 9.3 times (P < 0.0001), 11.2 times (P < 0.0001), and 6.1 times (P = 0.0051) compared to the miR-NC groups, respectively (Figure 5(a)). In other words, AFF4 showed the most significant binding with miR-1225-3p and was screened for subsequent experiments. TargetScan analysis showed that miR-1225-3p had two binding sites for AFF4 (Figure 5(b)). Targeting analysis revealed that the AFF4-WT, MUT1, and MUT2 groups showed decreased luciferase activity by 55% (P < 0.0001), 40% (P < 0.0001), and 25% (P = 0.0013), respectively, after miR-1225-3p mimic treatment compared to miR-NC combined with AFF4-WT, or MUT1, MUT2; the change in luciferase activity was not significant in the co-MUT group compared to miR-NC combined with co-MUT (P = 0.9823; Figure 5(c)). Moreover, the expression levels of AFF4 mRNA in keloid tissue and KFs were significantly upregulated compared to that in normal skin tissue (P < 0.0001) and NFs (P = 0.0001; Figure 5(d,e)).

**Figure 5.** miR-1225-3p targets AFF4. (a) RNA pull-down assay was performed to examine the enrichment of TRAM1, AFF4, KIF3B, MCHR1 and BICDL2 in keloid fibroblasts treated with Bio-miR-1225-3p. **P < 0.001 vs. Bio-NC. (b) Schematic diagram of h AFF4 and miR-1225-3p. (c) The relative luciferase activities were evaluated in HKFs after co-transfection with AFF4-WT, MUT1, MUT2, or co-MUT and miR-1225-3p mimic or miR-NC, respectively. **P < 0.001 vs. miR-NC. (d) The relative RNA levels of AFF4 were evaluated by qRT-PCR between keloid tissues (k) and normal skin (NS). **P < 0.001. (e) The relative RNA levels of AFF4 were evaluated by qRT-PCR between KFs and NFs. **P < 0.001 vs. NFs.

### Effects of miR-1225-3p on the survival and apoptosis of KFs via AFF4

To study the biological behavior of KFs accommodated by miR-1225-3p and AFF4, KFs were transfected with si-AFF4 or a miR-1225-3p inhibitor. Compared with the si-NC groups (P < 0.0001), knockdown of AFF4 reduced the expression levels of AFF4, which was abolished by the miR-1225-3p inhibitor (Figure 6(a,b)). CCK-8 and BrdU assays revealed that, contrast to the si-NC group, cell viability (P < 0.0001, at 48 h) and proliferation (P = 0.000) in the si-AFF4 group were inhibited, and the cell viability and proliferation induced by miR-1225-3p inhibitor were partially eliminated by AFF4 silencing (Figure 6(c,d)). Flow cytometry showed that AFF4 interference increased the level of apoptosis compared to that in the si-NC group (P < 0.0001), and miR-1225-3p inhibitor treatment reversed this effect (Figure 6(e)). Transwell analysis showed that the cell migration level was suppressed after transfection with si-AFF4 compared to that in the si-NC group (P < 0.0001), and the miR-1225-3p inhibitor alleviated the suppressive effect of si-AFF4 on migration (Figure 6(f)).

**Figure 6.** Effects of miR-1225-3p on the survival and apoptosis of KFs via AFF4. (a) The transfection efficiency of AFF4 mRNA was evaluated by qRT-PCR in KFs transfected with si-AFF4 or miR-1225-3p inhibitor. (b) The AFF4 protein level was evaluated by western blot in KFs transfected with si-AFF4 or miR-1225-3p inhibitor. (c) CCK-8 assays were performed to assess the viability in KFs transfected with si-AFF4 or miR-1225-3p inhibitor. (d) BrdU assays were performed to assess the proliferation ability in KFs transfected with si-AFF4 or miR-1225-3p inhibitor. (e) Cell apoptosis was examined using flow cytometry in KFs transfected with si-AFF4 or miR-1225-3p inhibitor. (f) Transwell migration assays were applied for assessing the migration ability of KFs transfected with si-AFF4 or miR-1225-3p inhibitor. *P < 0.05, **P < 0.001 vs. si-NC; ##P < 0.001 vs. si-AFF4+ inhibitor-NC.

## Discussion

Keloid formation is associated with skin trauma, inflammation, and increased wound tension [28]. Overactive fibroblasts produce large amounts of collagen and growth factors involved in the pathogenesis of keloids [3]. Furthermore, KFs exhibit higher proliferation and lower apoptotic rates than those observed in typical wound healing [29]. In addition, there is increasing evidence for the involvement of circRNAs in keloid regulation. For example, circ_101238 expression levels are upregulated in keloid tissues, stimulating cell growth by activating KF proliferation, while inhibiting apoptosis [30]. circNRIP1 knockdown successfully blocks the proliferation of KFs and expression of extracellular matrix proteins, while increasing the apoptosis rate [31]. In this study, we confirmed for the first time the effects of hsa_circ_0057452 on KF viability, migration, and apoptosis, and explored the specific mechanism by which hsa_circ_0057452 regulates keloid progression.

Shi et al. [13] constructed an interaction network of circRNA-miRNA-mRNA utilizing circRNA microarrays in keloids and found that these non-coding RNAs participate in keloid pathogenesis by influencing the cell cycle pathways. Similar mechanisms have been explored in subsequent studies. Lv et al. [32] found that circCOL5A1 released Epac1 as a competing endogenous RNA via adsorption of miR-7-5p to facilitate pathological hyperplasia of keloids. Zhang et al. [33] revealed that the interaction between hsa_circ_0001320 and miR-574-5p regulates the keloid pathology. In this study, we demonstrated that hsa_circ_0057452 is overexpressed in keloids, which is consistent with previously published circRNA microarray analysis [13]. In addition, functional experiments showed that hsa_circ_0057452 acts as a fibrosis promoter to augment the survival of KFs, while inhibiting apoptosis. A mechanistic analysis identified miR-1225-3p as a potential target of hsa_circ_0057452. Simultaneously, we found a significant decrease in miR-1225-3p expression levels in keloids. Moreover, low expression levels of miR-1225-3p promoted the malignant behavior of KFs and changed the effect of hsa_circ_0057452-silencing on cell function.

This study predicted AFF4 to be a target of miR-1225-3p via bioinformatics analysis. AFF4 levels were found to be significantly elevated in keloids. AFF4 is involved in the regulation of cancer cell proliferation, invasion, and survival in vitro, and tumorigenicity in vivo [34]. This suggests that AFF4 plays a positive role in cell survival. Similarly, AFF4-silencing inhibited the survival and metastasis of KFs, and induced their apoptosis. In addition, mechanical function experiments showed that AFF4 acted on keloid genesis and development via targeted inhibition by miR-1225-3p.

This study has several limitations. First, keloids need to be surgically removed within a limited time, resulting in a limited number of clinical samples. Moreover, there is a lack of animal models to study the effects of the hsa_circ_0057452/miR-1225-3p/AFF4 axis on keloids in vivo. Future research studies should expand the clinical sample size and use a nude mouse subcutaneous transplantation model with excised keloids for subsequent analysis.

## Conclusion

In conclusion, expression levels of hsa_circ_0057452 and AFF4 were found to be upregulated in keloids, while those of miR-1225-3p were downregulated. hsa_circ_0057452 promotes the proliferation and migration of KFs and inhibits their apoptosis by releasing AFF4 via sponging of miR-1225-3p. Our results shed light on the key role of hsa_circ_0057452 in keloid pathogenesis and may provide novel insights into the diagnosis and treatment of keloids.

## Supplementary Material

Supplemental Material

## Data Availability

The datasets used and/or analyzed during the current study are available from the corresponding author on reasonable request.https://circinteractome.nia.nih.gov/index.htmlhttps://www.targetscan.org/vert_71vv
